# A Review of Nanomaterials with Different Dimensions as Lubricant Additives

**DOI:** 10.3390/nano12213780

**Published:** 2022-10-27

**Authors:** Wenwen Liu, Xiaoxi Qiao, Shida Liu, Ping Chen

**Affiliations:** School of Mechanical Engineering, University of Science and Technology Beijing, Beijing 100083, China

**Keywords:** lubricating additives, nanomaterials, dimensions, tribological performance

## Abstract

Lubricant additives can effectively enhance the performance and environmental adaptability of lubricants and reduce the energy loss and machine wear caused by friction. Nanomaterials, as important additive materials, have an essential role in the research and development of new lubricants, whose lubrication performances and mechanisms are not only related to their physical and chemical properties, but also influenced by the geometric shape. In this paper, the friction reduction and antiwear performances of nanomaterials as lubricant additives are first reviewed according to the classification of the dimensions, and their lubrication mechanisms and influence rules are revealed. Second, the recent research progress of composite nanomaterials as lubrication additives is introduced, focusing on their synergistic mechanism to improve the lubrication performance further. Finally, we briefly discuss the challenges faced by nanoadditives and provide an outlook on future research. The review expects to provide new ideas for the selection and development of lubricant additives to expand the application of nanoadditives.

## 1. Introduction

Friction plays an important role in human production and life but, especially in industrial production, has consumed a large amount of primary energy. Lubrication failure and wear cause 80% of machine parts to fail [1]. The annual economic loss due to friction and wear in developed countries is 2–7% of their gross domestic product (GDP). The survey shows that China lost about CNY 4.95 trillion in 2019 due to friction and wear, accounting for 5% of GDP [2]. Therefore, using advanced lubrication technology is important for reducing friction and wear, saving energy, and reducing consumption in production and manufacturing [3,4]. At present, using lubricants is the most effective lubrication technology [5], which works by forming lubricating films between the friction surfaces to prevent their direct contact, thereby reducing the adverse effects of friction [6].

It is noteworthy that only using the lubricating oil as a lubricant is often challenging to achieve the ideal lubricating effect in some working conditions, and there may be problems, such as poor antiwear and limited friction reduction effect; meanwhile, it cannot satisfy some extreme working conditions, such as strong corrosion, strong oxidation, and strong reduction [7,8]. To further improve the performance of lubricants, a large number of lubricant additives are widely studied and applied. Lubricant additives are essential to maintain the overall performance of lubricants and can effectively improve the lubricating ability of the lubricant in boundary and hybrid lubrication states. It is also capable of manipulating specific characteristics, such as condensation, oxidation, blistering, and corrosion tendencies [9]. In boundary lubrication and hybrid lubrication states, as the lubricant fails to completely isolate the two friction surfaces and there is a considerable degree of direct contact between the friction surfaces, lubricant additives are required to protect the friction surfaces by specific chemical or physical means to reduce wear.

Numerous studies have shown that nanomaterials, such as metals [10], metal oxides [11], metal sulfides [12,13], and carbon nanomaterials [14,15,16], can greatly improve the friction reduction and antiwear properties due to their unique size, shape, and physicochemical properties [17,18]. According to their structural dimensions, nanomaterials are classified as zero-dimensional, one-dimensional, and two-dimensional nanomaterials (Figure 1). Zero-dimensional nanomaterials are materials that enter the nanoscale range in all three dimensions, two dimensions oriented to the nanoscale are one-dimensional nanomaterials, and two-dimensional nanomaterials have only one dimension oriented to the nanoscale. In various types of tribological applications, we are concerned that the shape of nanomaterials plays an important role in their lubrication performance and mechanisms, and can directly affect the contact pressure applied during loading. In addition, the nanoadditive package, with multiple nanomaterials in sympathetic action, provides better friction reduction and antiwear performance than a single nanoadditive [19].

In the paper, the nanomaterials as lubricant additives are classified and reviewed according to their structural dimensions. We discuss the lubrication performance and mechanisms and the main influencing factors of different dimensional lubricant additives. In addition, we review the research progress of different dimensional nanomaterials’ composite as lubricant additives and their synergistic effects in friction reduction and antiwear mechanism, explore the problems of commonly used lubricant additives, and prospect the future research of lubricant additives.

## 2. Single Nanoadditive

### 2.1. Zero-Dimensional Nanoadditive

Zero-dimensional nanoadditives mainly include clusters and nanoparticles. The representative material of the cluster is fullerene (C_60_), which is a stable spherical structure with a diameter of about 0.7 nm. It has high mechanical strength, higher pressure resistance than diamonds, and a microhardness of up to 18 GPa [20,21,22,23]. Nanoparticles refer to ultrafine particles of nanometer scale, which are larger than atomic clusters, generally within 100 nm. The representative materials are metal and its oxide nanoparticles, such as Cu, Fe, Ag, Al_2_O_3_, TiO_2_, and ZnO.

At present, the lubrication mechanisms of zero-dimensional nanomaterials as additives mainly include three aspects (Figure 2): (1) the spherical structure of nanoparticles can achieve the effect of “rolling bearing”, in which the rolling body is the ball, so as to reduce the friction resistance, as shown in Figure 2a; (2) nanoparticles have a small particle diameter in the nanoscale, and then it can fill the scars and grooves on the friction surfaces, repairing the surface mechanical damage, as shown in Figure 2b; (3) nanoparticles under specific conditions can form a protective film on the friction surfaces, which in turn reduces the degree of mechanical wear, as shown in Figure 2c. It is recommended that specific working conditions are required to achieve the above three lubrication mechanisms, in practice; it may be one or more of the lubrication mechanisms. Generally, the “rolling bearing” effect can work at smaller loads when the thickness of the lubricant film is comparable to the diameter of the nanoparticles [24]. At high temperatures and high contact stress conditions, zero-dimensional nanomaterials are more likely to form protective films on the surfaces.

Kumara et al. [25] found that the oil-soluble Ag nanoparticles almost did not affect the lubricating performance of poly-alpha-olefin (PAO) base oil in the mixed lubrication condition, because the contact pressure was insufficient to produce a silver deposit layer in the contact area and no “rolling bearing” effect was formed. However, under the boundary lubrication conditions, the Ag nanoparticles can form a 50–100 nm thick silver-rich protective film between the friction surfaces, and the organic molecules modified on the particle surfaces made themselves strongly adsorb on the positively charged metal surfaces, achieving 35% and 85% reduction in friction coefficient and wear amount compared with the neat PAO base oil, respectively.

The improvement effect of nanoparticles as lubricant additives on lubrication performance is related to the viscosity of lubricants. High viscosity will limit the rolling effect. Ku [26] and Lee et al. [27] found that C_60_ did not significantly improve the lubrication performances of lubricant oil with high viscosity. However, it has a significant effect on improving the tribological properties of lubricant oils with low viscosities. Additionally, the improvement effect is influenced by the lubricant polarity. The addition of nanoparticles may deteriorate the uniform and good adsorption of polar oils on the metal surfaces, and the lubricant polarity promotes the aggregation of nanoparticles, which hinders the formation of nanoparticle films. Meanwhile, the agglomerated nanoparticles may lead to three-body abrasive wear between the friction surfaces, increasing the friction coefficient and wear loss. Guzman Borda et al. [28] showed that Cu nanoparticles did not improve and enhance the antiwear properties of the polar synthetic ester-based oil. In contrast, the addition of Cu nanoparticles to nonpolar mineral oil reduced the friction coefficient by 60% and the wear amount by 60%.

The hardness and shear modulus of the nanoparticles also affect the degree of enhanced lubrication performance. Zhang et al. [29] carried out a study on the enhanced lubrication properties of Sn and Fe nanoparticles with multialkylated cyclopentane (MAC) under vacuum conditions. Results showed that both kinds of nanoparticles could form protective films with low shear resistance and hardness on the friction surfaces. However, compared with Sn nanoparticles, Fe nanoparticles are more effective in antiwear, but have relatively poor cooling and friction reduction effects due to the higher hardness and higher shear modulus, as well as the better compatibility and more stable bonding between the Fe protective film and the frictional steel ball surface. On the contrary, Sn nanoparticles are more effective in reducing the friction coefficient but less effective in antiwear.

Additionally, the stability of protective films formed by nanoparticles during friction is very critical [30,31]. Ingole et al. [31] showed that due to the repulsive forces between the nanoparticles and lubricant molecules, the oleophobic TiO_2_ nanoparticles can be deposited on the friction surfaces and form a uniform and stable protective film, which can effectively stabilize the friction coefficient of the mineral oil, although it has limited effect in reducing the friction coefficient.

The dispersibility of nanoparticles in lubricants is the key to their effectiveness in improving lubrication performance. On the one hand, good dispersion stability can ensure that nanoparticles enter the friction interface more easily. Luo et al. [32] found that hydrophobically modified Al_2_O_3_ nanoparticles can effectively prevent agglomeration under the effect of electrostatic repulsion, which led to good dispersion stability in the lubricant and enabled the nanoparticles to maintain a small size to enter the friction surface easily. Under the action of contact pressure, Al_2_O_3_ nanoparticles formed a self-laminating film on the friction surfaces to repair the surface furrow. Meanwhile, the spherical structure of Al_2_O_3_ nanoparticles can transform sliding friction into rolling friction, which significantly improves the friction reduction and antiwear performance. On the other hand, the aggregation of nanoparticles can lead to clogging of the lubricant and deterioration of the lubrication effect, so researchers have been trying to improve the dispersion stability of nanoparticles in lubricants to enhance the lubrication performance.

Carbon quantum dots (CQDs) are a class of zero-dimensional carbon nanomaterials with remarkable fluorescence properties, whose surfaces are filled with a large number of hydroxyl and carboxyl groups [33]. CQDs have good dispersion and stability, adjustable surface functional groups, low toxicity, and environmentally friendly properties, but their texture is softer than fullerenes and can be easily compressed into laminar structures. Xiao et al. [34] prepared a kind of water-soluble CQD nanomaterial as a lubricant additive to improve the lubrication performance of deionized water. Results showed that under certain work conditions, most of the CQDs provided a “rolling bearing” effect at the beginning of the friction experiments. Along with the test, the normal stress and shear stress crushed part of the CQDs, generating a laminar structure for shear sliding. If adding a high concentration of CQDs, it takes longer to crush them, so the rolling effect lasts longer and the lower friction coefficient can last longer.

In conclusion, it is crucial point how to make the best use of the “rolling bearing” effect of zero-dimensional nanomaterials to improve the lubrication performance. Additionally, the lubrication performance of zero-dimensional nanomaterials is closely related to working load and velocity, the physical and chemical properties of nanoparticles and lubricant (such as hardness and shear modulus of nanoparticles and polarity and viscosity of lubricants), dispersibility of nanoparticles, and direct interaction between nanomaterials and lubricants (or friction surfaces). Compared with metal nanoparticles, metal oxides are more stable and are more likely to form stable boundary lubrication films on friction surfaces under boundary lubrication conditions, thus improving lubrication performance.

### 2.2. One-Dimensional Nanoadditives

One-dimensional nanomaterials include nanorods, nanotubes, and nanofibers with high aspect ratios. Common one-dimensional materials include carbon nanotubes (CNTs) and one-dimensional metal compound additives, such as CuS, WS_2_, ZnO, and MoS_2_ [35].

The lubrication mechanisms of one-dimensional nanomaterials as additives are similar to those of zero-dimensional nanomaterials, mainly including the “rolling bearing” effect (Figure 3), the film-formation mechanism, and the effects of filling and repairing the scars and grooves. The difference is that the “rolling body” in the “rolling bearing” effect of one-dimensional nanomaterials is a cylindrical roller.

CNTs are tubular structures composed of carbon atoms arranged in a hexagonal pattern [36], which have excellent thermal and mechanical properties and good self-lubricating performance [37]. According to the number of tube walls, CNTs can be classified into single-wall carbon nanotubes (SWCNTs) and multiwall carbon nanotubes (MWCNTs). The high thermal conductivity of CNTs can resist frictional heat and reduce surface temperature and intersurface adhesion [38]. Compared with SWCNTs, MWCNTs have better thermal conductivity and more applications.

Khalil et al. [39] found that MWCNT films deposited on worn surfaces can reduce the direct metal surface contact and decrease the shear stress, which improved the wear resistance and load-carrying capacity of Mobil gear 627 and paraffinic mineral oil. Gong et al. [40] studied the effect of MWCNTs on the lubrication performance of polyalkylene glycol (PAG). Results indicated that when the load was 100 N, 0.08 wt% of MWCNTs could form a boundary lubricating film and thus significantly improve the friction reduction and wear resistance of PAG. However, when the load was increased to 125 N, MWCNTs’ boundary film was destroyed under the effects of high temperatures and high loads; thus the friction coefficient suddenly increased and stabilized at a value comparable to that of pure PAG.

As we know, the dispersity of nanoadditives is critical for improving lubrication performances. However, because of the chemical inertness and high surface energy of CNTs, they are highly prone to agglomeration, so most studies have used functionalized modifications to improve their dispersion stability and thereby lubrication performance. Cornelio et al. [41] studied the lubrication performance of COOH-functionalized CNTs and found that the polar functional group not only improved the CNTs’ dispersion stability, but also facilitated the adsorption of CNTs on friction surfaces, and thus can effectively reduce the friction coefficient and wear rate of both oil and water systems. Kumar et al. [42] also used COOH -functionalized MWCNTs, which effectively improved the lubricity properties of polyalphaolefin (PAO100) and polypropylene glycol (PPG 2000). In the initial test phase, the friction protective film was not formed and the addition of MWCNTs deteriorated the lubricity of the lubricant oil instead. However, as the friction progressed, the formed MWCNTs’ protective film and the “rolling bearing” effect caused by their orderly arrangement in the contact area began to work, showing excellent lubricity for a longer period. It is worth noting that when the contact pressure of friction pairs is too high, MWCNTs may be compressed into layers, thus reducing the “rolling bearing” effect.

Researchers also have fabricated metal compounds into one-dimensional nanotubes or nanorods as lubricant additives. Zhang et al. [43] found that WS_2_ nanorods as a lubricant additive exhibit good friction reduction and antiwear properties with both friction film and “rolling bearing” effects. Rajkumar et al. [44] showed that 0.02 wt% of ZnO nanorods significantly reduced the friction coefficient of SAE (20W-40) engine oil by about 27.6%. The better lubrication performance compared with spherical ZnO nanoparticles is due to the fact that ZnO nanorods have a larger contact area and are subjected to the weaker shearing action of the lubricating fluid, resulting in a higher binding ability to the surface. Chen et al. [45] found that CuS nanorods effectively enhanced the lubricating performance of liquid paraffin waxes mainly due to the deposition of CuS on friction surfaces to form a friction protective film, and the oleic-acid-modified CuS nanorods had higher dispersion stability, which allowed them to easily enter the contact interface with minimal agglomerate size, forming a more uniform and complete friction film, resulting in 50% and 10% reductions in friction coefficient and wear rate, respectively, relative to the addition of unmodified CuS. 

Nanotubes made of metal compounds have a lower strength compared with nanorod structures. Meanwhile, they have higher plasticity and ductility than CNTs and can easily form a friction-protective film with low shear resistance under high loads. Wu et al. [46] found that MoS_2_ nanotubes maintain better friction reduction performance at higher loads and rotational speeds, because MoS_2_ nanotubes are compressed into nanosheets during friction, and the larger the spread area of the nanosheets, the lower the friction coefficient.

In summary, for one-dimensional nanomaterials, one important point is to convert the sliding friction to rolling friction as much as possible; thus it is necessary to pay attention to the orientation of one-dimensional nanomaterials [47]. In the case of CNTs, the “rolling bearing” effect is related to the nature of lubricants and the friction pairs, working conditions, and dispersion stability. The agglomeration of CNTs can block lubricants and thus deteriorate the lubrication performance [48]. Unlike the dominant role of CNTs’ “rolling bearing” effect, the friction reduction and antiwear performance of one-dimensional metal compounds generally depend on the formation of friction-protective films under high stress. Therefore, increasing the concentration of metal compounds to a certain extent is beneficial for forming more uniform and complete protective films to improve lubrication performance [43,44,45,46,47,48,49].

### 2.3. Two-Dimensional Nanoadditives

Two-dimensional nanomaterials as lubricant additives have the advantages of an ultrathin lamellar structure, low shear strength, high specific surface area, and excellent mechanical and self-lubricating properties [50]. Typical commonly used two-dimensional nanoadditives include graphene and its derivatives [51,52,53,54], hexagonal boron nitride (h-BN) [55], molybdenum disulfide (MoS_2_) [56], and MXene [57]. Different two-dimensional nanomaterials have different layer spacing (Table 1), and the layer spacing has a great effect on the lubrication performance.

The excellent self-lubricating properties of two-dimensional nanomaterials are related to their in-plane strong bonding and interlayer weak interaction. In-plane strong bonding makes the formed monolayer with high modulus and high strength, and interlayer weak interaction results in easily sliding between layers. Furthermore, the high specific surface area makes it easy to adsorb to the friction surface to form a protective film. Therefore, in addition to the same mechanisms of forming friction protection film and filling grooves to repair surface lubrication as zero/one-dimensional nanomaterials, another key factor for two-dimensional nanomaterials to improve the lubrication performance is the interlayer sliding behavior with low shear strength (Figure 4).

The interlayer sliding behavior of two-dimensional nanomaterials is closely related to their nanostructures. Zhao et al. [62] found that the original exfoliation degree of graphene plays a key role in the evolution of its nanostructure. As shown in Figure 5, graphene with a higher degree of exfoliation can be restacked into a laminar friction film parallel to the sliding direction under the pressure and shear of the friction pair, and interlayer sliding occurs, which leads to better lubrication performance.

Graphene oxide (GO), an important graphene derivative, consists of the graphene backbone with many oxygen-containing groups on both the basal plane and the edges. Due to the good hydrophilicity of these groups, including hydroxyl, carboxyl, and epoxy groups, GO is more suitable than graphene as a water-based lubricant additive. The introduction of oxygen-containing groups in GO provides a large number of active sites for surface modification, which gives it the advantages of easy functionalization and high controllability [63,64]. Additionally, different C/O ratios of GO can affect its lubrication performance. Cheng et al. [65] found that graphene with a lower C/O ratio was more easily dispersed in basic oil and more readily adsorbed on the friction surfaces to form protective films, improving the friction reduction and antiwear ability of GO.

However, excessive oxygen-containing groups in GO may restrict interlayer sliding [63], so the application of reduced graphene oxide (RGO), which can be obtained by removing part of the oxidized functional groups through chemical reduction, has attracted the attention of researchers. Zhao et al. [63] found that RGO can significantly reduce the friction coefficient of PAO6 by about 30%, and the friction chemical reaction film of RGO is more robust and stable. Meanwhile, GO with different concentrations only slightly reduces the friction coefficients of PAO6, and the friction coefficient instability is much greater than that of PAO6 doped with RGO.

Research shows that the morphological regularity of graphene will also directly affect its lubricating performance. Mao et al. [66] investigated the lubrication performance of three types of reduced graphene oxide sheets with different micromorphologies, including those with regular edges (RG), irregular edges (ir-RG), and both irregular edges and wrinkles (ir-RWG), as shown in Figure 6. Results showed that RG with regular edges could form a thick, firm, and continuous friction film and obtained excellent lubrication performance. In contrast, ir-RG and ir-RWG only formed a thin and broken friction film, which even hindered the sliding.

The interlayer interaction strength of two-dimensional nanomaterials is also essential in improving the lubricity. Fluorinated graphene (F-Gr), as a graphene derivative, has different layer spacings and interlayer interaction forces with graphene due to the introduction of fluorine atoms [67]. Hou et al. [68] investigated the tribological properties of F-Gr with three different fluorine element contents. Results showed that F-Gr with higher fluorine content has larger layer spacing, weaker interlayer van der Waals forces, and larger relative interlayer slip under shear stress, which can significantly reduce wear and the friction coefficient. In addition, the introduction of fluorine atoms can improve the adsorption of F-Gr on the metal surface. Chen et al. [69] showed that F-Gr adsorbed more easily than graphene on the friction surfaces to form a protective film, which better improved the lubricity of PAO6.

The application of graphene as a lubricating additive also faces the dispersion problem, which can be improved by changing the physical morphology, chemical modification, and dispersants. Li et al. [70] produced highly exfoliated RGO by thermal reduction to enhance the specific surface area and stable dispersion in PAO6 for up to 4 days. Yu et al. [71] modified GO with octadecylamine (ODA) via amidation and made GO stably dispersed in Shell series GTL8 base oil for about 2 weeks. Wu et al. [72] used chemically modified graphene (0.5 wt%) and a dispersant (1 wt%) in combination to maintain stable dispersion in PAO6 for up to about 120 days.

MoS_2_ is also an important two-dimensional nanomaterial [73] with a reliable lubricating capacity over a wider temperature range compared with graphene. In addition, MoS_2_ has better tribological properties in anaerobic environments [74]. Zhao et al. [75] revealed that the sulfur element of MoS_2_ can easily react with the friction surfaces to form sulfides or even sulfates, promoting more stable adsorption of molybdenum disulfide. In contrast, the graphene friction film had poor adsorption properties and stability, and was more prone to breakage. Thus, although both materials can form boundary adsorption films, MoS_2_ had better lubricating properties than graphene. More importantly, the excellent adsorption performance of MoS_2_ is not affected by surface roughness. Wang et al. [56] achieved good dispersion stability of MoS_2_ in water by thiol modification, and the good dispersion ensured that MoS_2_ could continuously exist between contact surfaces and adsorb on friction surfaces, thus achieving the purpose of protecting friction surfaces and reducing wear.

h-BN, also known as “white graphite”, has better antioxidant and anticorrosion properties than graphene [76]. Like other two-dimensional nanomaterials, h-BN as a lubricant additive has the function of filling repair [77] and interlayer sliding. Meanwhile, it can generate a boron oxide (B_2_O_3_) friction chemical film by friction chemical reaction. Abdollah et al. [78] found that h-BN can significantly improve the lubricating properties of pure water, and the appropriate increase in h-BN concentration can change the lubrication state of water-based lubricants from mixed lubrication to hydrodynamic lubrication. Ma et al. [79] successfully exfoliated a flake nanosheet h-BN with 100 nm ultrathin thickness from a block h-BN and compared the effects of the two forms of h-BN on the lubricating properties of base oils. The results showed that the nanosheet structure of h-BN was easier to cover the friction surface and form a lubricating protective film due to its larger specific surface area. Therefore, the effect of the sheet structure of h-BN on friction reduction and antiwear was better than that of the block h-BN.

MXene, a series of transition metal carbides or nitrides with strong interfacial coupling properties compared with carbon-based nanomaterials, is capable of forming strong self-lubricating transfer films [80]. In particular, MXene has good heat resistance, which can still be in excellent lubrication conditions at several hundred degrees Celsius [81]. Yi et al. [82] adopted molybdenum carbide (Mo_2_CT_x_) MXene as the additive of lithium hexafluorophosphate-based ionic liquid, which achieved the superlubricity state with a friction coefficient of 0.004 between silicon nitride and sapphire friction pairs with the maximum contact pressure up to 1.42 GPa, far exceeding the pressure limit of the superlubricity in previous studies. The excellent lubrication performance is the result of the combined effects of very low interlayer shear strength of (Mo_2_CT_x_) MXene and the composite friction film (containing mainly molybdenum oxide and phosphorus oxide) produced by friction chemical reactions.

In conclusion, for two-dimensional nanomaterials to improve the lubrication performance, the key point is to enhance the interlayer sliding behavior and reduce the friction resistance. Meanwhile, the interlayer sliding behavior is mainly influenced by many factors, such as morphological regularity, surface active groups, stacking, defects, layer spacing, the number of layers, and so on. For example, graphene nanosheets without obvious defects have better lubrication performance than those with some original structural defects, such as dislocations and vacancies [83]. 

Here, we summarize some studies on the tribological performance of nanomaterials with different dimensions as lubricant additives, as shown in Table 2. Relevant experimental studies have shown that single nanoadditives have good tribological effects. Besides, other studies have shown that there may also be an synergistic effect between different nanomaterial lubrication additives, and the composite nanoadditives with a synergistic effect of two or more nanomaterials can make up for the defects of single nanoadditives and obtain better wear reduction and friction reduction performance.

## 3. Composite Nanoadditives

Composite nanoadditives are additives containing two or more kinds of nanomaterials, which can be of the same or different dimensions. In addition to using their respective advantages, composite nanoadditives may also have synergistic effects under certain matching conditions and exhibit more excellent lubricating properties [84]. Making full use of the synergistic lubrication mechanism of multiple nanoadditives is the key to further developing excellent lubricants. 

Kim et al. [85] found that hydrophilic zero-dimensional nanodiamond (ND) can be uniformly dispersed between graphene sheet layers, reducing interlayer interaction forces and promoting interlayer sliding. Meanwhile, the zero-dimensional ND can reduce the stress concentration and improve the mechanical flexibility of graphene, which in turn effectively improves the lubrication performance. 

Wang et al. [86] fabricated composite lubrication additives, including zero-dimensional copper perrhenate Cu(ReO_4_)_2_ nanoparticle and graphene, which can adapt to lubrication in a wide temperature range. When the temperature is lower than 300 °C, graphene plays the main lubricating role; when the temperature is higher than 300 °C, a formed mixed layer, which contains the bimetallic oxide Cu(ReO_4_)_2_ and the residual carbides produced by graphene, acts as the hard phase to improve the bearing capacity of the lubricating layer. Furthermore, the thermal softening effect of Cu(ReO_4_)_2_ can improve the plasticity of the mixed layer and reduce surface wear caused by hard particles. The friction coefficient of PAO6 can be significantly reduced by 62.4% at 500 °C with 0.05 wt% of the composite lubricant additive. 

Meng et al. [87] uniformly anchored Ag nanoparticles on the outer wall of MWCNTs by aldehyde reduction, and adding 0.18 wt% of the Ag/MWCNTs nanocomposite to 10w40 engine oil can reduce the friction coefficient by 36.4% and the wear scar diameter (WSD) by 32.4%. Throughout the friction process, Ag/MWCNT nanocomposite shows better lubrication performance than either Ag nanoparticles or MWCNTs alone. Meanwhile, the study found that Ag/MWCNTs’ nanocomposite can reduce friction and wear by filling the grooves and forming a physical deposition film on the wear surface. The high load-bearing capacity and high thermal conductivity of MWCNTs can facilitate the formation of a continuous oil film during the friction process, while a large number of Ag nanoparticles were released on the friction surface to continue the friction-reducing effect.

In addition to the composite nanoadditives formed by mixing different nanomaterials, they can also be generated by chemical methods with various nanomaterials. Wang et al. [88] modified Ag nanoparticles with CQDs as the lubricant additive of PAO6. Results showed that PAO6 doped with Ag-CQDs’ nanocomposites reduced the friction coefficient by 13.4% over that of PAO6 doped only with CQDs’ nanoparticles. This is because the Ag nanoparticles can improve the thermal stability of the CQDs’ friction film formed during the friction process, which can adapt to higher temperatures. Additionally, the hardness of Ag is higher than that of CQDs, which improves the load-bearing capacity of the friction film. 

Additionally, heterogeneous structures formed chemically by two-dimensional nanomaterials with different lattices can produce ultralow friction. Kumari et al. [89] synthesized h-BN/MoS_2_ heterostructures by growing MoS_2_ flakes in h-BN nanosheets through the chemical reduction method in a cetyltrimethylammonium bromide (CTAB) environment. The addition of a microdose (30 ppm) to engine oil achieved an ultralow friction coefficient of 0.067. Compared with pure 5W30 engine oil, the coefficient of friction and wear were reduced by 77.5% and 90%, respectively. On the one hand, the synergistic effect of the two different two-dimensional nanomaterials reduces the agglomeration and improves the dispersion performance. On the other hand, the asymmetric stacking of h-BN and MoS_2_ makes the interlayer sliding easier. Due to the good adsorption ability of MoS_2_ on the metal surface, it is easier for the heterogeneous structure to form protective films on the steel friction interface. The heterostructures are expected to be developed as a revolutionary material for a new generation of lubricants. 

## 4. Conclusions and Outlook

In summary, due to the unique dimensional structure and physical and chemical properties, nanomaterials as lubricant additives can significantly improve the lubrication performance through a proper design. The lubrication mechanisms of nanomaterials include the film-formation mechanism, mending or self-repairing effect, and “rolling bearing” or “interlayer sliding” mechanisms related to the dimensionality of nanomaterials. The friction protective films can be formed by physical or chemical methods, such as deposition films, physical or chemical adsorption films, and chemical reaction films. Additionally, surface adsorption strength, distribution uniformity, and thickness of the friction-protective films will affect their friction reduction and antiwear performance. For example, the sulfur elements of MoS_2_ nanoparticles can react with the metal surface to form a chemical reaction film with higher bond strength, which can better improve the wear resistance of the friction pairs. Mending or self-repairing effect means that nanomaterials can fill the wear scars and grooves on friction surfaces due to their small size to repair the worn surface and reduce wear. The “rolling bearing” or “interlayer sliding” mechanism is related to the dimensionality of nanomaterials, where zero- and one-dimensional nanomaterials can form a “rolling bearing” effect, turning sliding friction into rolling friction. Furthermore, the weak interlayer interaction of two-dimensional nanomaterials leads to “interlayer sliding”, which reduces the shear resistance between the friction pairs. Therefore, in the design of high-performance lubricant additives, both the physical and chemical properties of nanomaterials and their lubrication mechanisms should be considered to realize the regulation and optimization of lubrication performance (Table 3).

At high loads and high speeds, materials with high modulus of elasticity can well separate the two metal surfaces and easily form a “rolling bearing” lubrication mechanism. However, when the load is too high, the nanoadditive will become abrasive particles and cause furrows on the surface. Materials with high plasticity and ductility adapt to high-pressure and high-speed environments by forming a protective film that can be easily sheared. At low loads, if the oil film thickness is comparable to the diameter of the nanomaterial, a “rolling bearing” effect is easily formed. Highly thermally conductive materials are more adaptable to high-temperature environments and can easily form protective film mechanisms. It is necessary to consider the viscosity of lubricating oil, the hardness of nanomaterials and friction pairs, and the working load and speed to better realize the “ball bearing” effect in the zero-/one-dimensional nanomaterial lubrication design. In addition to the factors mentioned above, alignment orientation is also a key factor to be considered in achieving the “rolling bearing” effect for one-dimensional nanomaterials. For the “interlayer sliding” effect of two-dimensional nanomaterials, the interlayer interaction strength should be paid much attention to. For composite nanomaterials as lubricant additives, it is expected to synergize their respective advantages to achieve better performance than a single nanoadditive, thus improving the lubrication performance.

With the urgent need to save energy and resources, research on superlubricity and ultralow wear has become the latest trend in tribology. Meanwhile, with the development of industry, more and more mechanical devices need to operate in extreme environments, such as high temperature, extreme pressure, high speed, heavy load, and high vacuum in marine or aerospace fields. Therefore, there is an urgent need to develop lubricants with nanomaterials as additives and reasonably designed nanoadditive packages composed of two or more nanomaterials in synergy to adapt to extreme operating conditions, while expecting to achieve superlubricity.

However, the application of lubricant additives faces some challenges. One of the most important is the dispersion stability of the lubricant additive. Good dispersion performance can ensure easier access of nanomaterials to the frictional contact zone and reduce clogging and lubrication deterioration caused by aggregation. Therefore, various modification techniques should be investigated to improve the dispersion stability of lubricant additives. In addition, it is worth noting that the addition of high concentrations of additives increases the viscosity of the base lubricant. Therefore, when adding nanoadditives to base lubricants, their physicochemical properties must be controlled within appropriate limits. Moreover, the high production cost of nanomaterials is also a significant challenge. Therefore, the production process of nanomaterials also needs to be optimized to improve the economic applicability of nanoadditives. 

In conclusion, it is still the focus of future research on using nanomaterials as lubricant additives, especially composite nanomaterials, to achieve high-performance lubrication under different working conditions. There is still no fully clear and unified theoretical guidance for that.

## Figures and Tables

**Figure 1:** Schematic of the carbon nanomaterials in different dimensions: (**a**) zero-dimensional fullerene, (**b**) one-dimensional carbon nanotubes, (**c**) two-dimensional graphene.

**Figure 2:** Diagram of the lubrication mechanism of zero-dimensional nanoadditive: (**a**) “rolling bearing” effect, (**b**) mending effect, (**c**) film-formation mechanism.

**Figure 3:** The “rolling bearing” effect of one-dimensional nanomaterials.

**Figure 4:** Interlayer slip mechanism of two-dimensional nanomaterials.

**Figure 5:** Schematic demonstration of the lubrication mechanism of the structural evolution of graphene additives. Reprinted with permission from [62]. © 2017 Elsevier B.V. All rights reserved.

**Figure 6:** (**a**–**c**) SEM; (**d**–**f**) TEM micromorphological images of the three types of graphene sheets: (**a**,**d**) for RG; (**b**,**e**) for ir-RG; (**c**,**f**) for ir-RWG. Reprinted with permission from [66]. © 2017 Elsevier Ltd. All rights reserved.

**Table 1:** Layer spacing of common two-dimensional nanomaterials.

Two-Dimensional Nanomaterials	Layer Spacing	Reference
Graphene	About 0.335 nm	[58]
Hexagonal boron nitride	About 0.333 nm	[59]
Molybdenum disulfide	About 0.65 nm	[60]
MXene	About 1.23–1.40 nm	[61]

**Table 2:** Tribological performance of nanomaterials with different dimensions as lubricant additives.

Dimensions of Nanoadditives	Nanomaterials	Lubricant	Optimal Concentration (wt%)	Operating Condition	Effect		Major Mechanism	Reference
					Antiwear	Friction Reduction		
Zero dimension	C_60_	Refrigerant oil	0.1	1000 rpm; 1200 N; GC200 disk-on-GC200 disk	-	33%	“Rolling bearing” effect; film-formation mechanism	[26]
	Cu	Paraffinic mineral	0.3	0.6 m/s; 588 N; AISI 1020 pin-on-AISI 52100 disk	64%	60%	Film-formation mechanism; mending or self-repairing effect	[28]
	Ag	PAO base oil	0.38	0.5 m/s; 100 N; AISI 52100 steel ball-on-A2 tool steel disk	85%	35%	Film-formation mechanism; “rolling bearing” effect	[25]
	Fe	MAC	0.2	1450 r/min; 300 N; AISI 52100 four-balls	-	25%	Film-formation mechanism; mending or self-repairing effect	[29]
	Al_2_O_3_	Base oil	0.1	1450 r/min; 147 N; GCr15 four-balls	41.75%	23.92%	Film-formation mechanism; “rolling bearing” effect	[32]
	CQDs	Deionized water	0.25	1.5 m/min; 2 N; Si_3_N4 ball-on-Si_3_N_4_ disk	-	30%	“Rolling bearing” effect; film-formation mechanism	[34]
One dimension	CNTs	PAG	0.08	3 m/min; 50 N; AISI 52100 ball-on-AISI 52100 disk	-	57%	Film-formation mechanism	[40]
	ZnO nanorod	SAE(20W-40)	0.02	1200 rpm; 400 N; AISI E52100 four-balls	-	27.6%	“rolling bearing” effect	[44]
	CuS nanorod	Liquid paraffin	2	300 rpm; 300 N; Pig iron pin-on-bearing steel disk	10%	50%	Film-formation mechanism	[45]
	MoS_2_ nanorod	150 SN base oil	0.08	1200 rpm; 100N; GCr15 four-balls	35%	39.2%	“Rolling bearing” effect; film-formation mechanism	[46]
Two dimension	Graphene	PAO6	0.5	0.144 m/min; 2 N; AISI 52100 ball-on-AISI 52100 disk	-	50%	Interlayer sliding	[62]
	RGO	PAO6	0.5	0.144 m/min; 2 N; GCr15 ball-on-GCr15 disk	-	30%	Interlayer sliding; film-formation mechanism	[63]
	F-Gr	PAO6	1	10 mm/s; 50 N; bearing steel ball-on-GCr15 steel disks	12.30%	87%	Film-formation mechanism	[69]
	MoS_2_	Hydraulic oil	0.1	2.4 mm/s; 3 N; GCr 15 ball-on-H62 brass disk	_	82%	Film-formation mechanism	[75]
	h-BN	Mineral lube	0.06	1200 rpm; 100 N; four-balls	35.20%	35.70%	Interlayer sliding; film-formation mechanism	[79]
	MXene	Lithium hexafluorophosphate-based ionic liquid	0.166	1200 rpm; 392 N; AISI 52100 four balls	-	92%	Film-formation mechanism	[82]

**Table 3:** Lubrication mechanism of nanolubricant additives in different dimensions.

Dimensions of Nanoadditives	Lubrication Mechanisms	
Zero dimension	“Ball roller bearing” effect	Film-formation mechanism and mending or self-repairing effect
One dimension	“Cylindrical roller bearing” effect	
Two dimension	Interlayer sliding	

## Data Availability

Not applicable.
